The article "Comparison of the Effects of Epidural Anesthesia and General Anesthesia on Perioperative Cognitive Function and Deep Vein Thrombosis in Patients Undergoing Total Knee Arthroplasty" was retracted in 2023. Reasons: unreliable results or conclusions; concerns about the data; concerns about the peer review; concerns about the citations.

# Comparison of the Effects of Epidural Anesthesia and General Anesthesia on Perioperative Cognitive Function and Deep Vein Thrombosis in Patients Undergoing Total Knee Arthroplasty

**DOI:** 10.1155/2021/1565067

**Published:** 2021-10-15

**Authors:** Zhenyu Wu, Yan Zhu

**Affiliations:** ^1^Department of Anesthesiology, Qinhuangdao First Hospital, Qinhuangdao, Hebei 066000, China; ^2^Department of Operation, Qinhuangdao First Hospital, Qinhuangdao, Hebei 066000, China

## Abstract

**Objective:**

To explore the effects of epidural anesthesia and general anesthesia on perioperative cognitive function and deep vein thrombosis (DVT) in patients undergoing total knee arthroplasty (TKA).

**Methods:**

Total of 68 patients undergoing TKA in our hospital from September 2019 to March 2021 were selected and divided into the control group under general anesthesia and the observation group under epidural anesthesia according to the different anesthesia methods, 34 patients in each group. TKA was selected in both groups and performed by the same group of physicians, anesthesiologists, and nursing staff. The mean arterial pressure (MAP), heart rate (HR), and blood oxygen saturation (SpO_2_) were observed immediately before anesthesia (T1), 30 min after anesthesia (T2), after surgery (T3), and 1 d after surgery (T4). The changes of platelet (PLC), fibrinogen (Fbg), prothrombin time (PT), activated partial thrombin time (APTT), and other coagulation indicators were recorded. The Montreal Cognitive Assessment (MoCA) scores before surgery and 1 d and 3 d after surgery were observed. The blood samples of the two groups were collected before surgery and 1 d and 3 d after surgery, and the levels of brain-derived neurotrophic factor (BDNF) and nerve growth factor (NGF) in the peripheral blood of the two groups were measured by ELISA. The number of postoperative mental disorders and DVT in the two groups was calculated.

**Results:**

The MAP and HR of T4 were lower than those of T1, T2, and T3. The MAP of T2, T3, and T4 in the observation group was lower than that in the control group (*P* < 0.05), and the SpO_2_ of T1–T4 in the two groups did not change significantly, and there was no significant difference between the two groups (*P* > 0.05). Compared with T1, there was no significant difference in PLC, Fbg, and PT in the observation group T4 (*P* > 0.05), and APTT was lower than T1 (*P* < 0.05). The PLC, PT, and APTT of T4 in the control group were all lower than those of T1 (*P* < 0.05), and there was no significant difference between Fbg and T1 (*P* > 0.05). The PLC, Fbg, and PT of T4 in the observation group were higher than those in the control group, while APTT was lower than that in the control group (*P* < 0.05). The MoCA scores of patients in both groups on the 1st and 3rd day after operation were lower than those before operation, and the observation group was higher than that in the control group (*P* < 0.05). The BDNF and NGF of patients in both groups were lower than those before operation on the 1st day after operation, and the BDNF and NGF in the observation group were higher than those in the control group on the 1st and 3rd day after operation (*P* < 0.05). The mental disorder (2.94%) and DVT incidence (2.94%) in the observation group were lower than those in the control group (29.41%, 26.47%) (*P* < 0.05).

The article "Comparison of the Effects of Epidural Anesthesia and General Anesthesia on Perioperative Cognitive Function and Deep Vein Thrombosis in Patients Undergoing Total Knee Arthroplasty" was retracted in 2023. Reasons: unreliable results or conclusions; concerns about the data; concerns about the peer review; concerns about the citations.

**Conclusion:**

Epidural anesthesia for patients with TKA can obtain better clinical effects, maintain stable hemodynamic and coagulation states, reduce stress response of patients at the same time, and reduce perioperative cognitive dysfunction and the incidence of DVT in patients.

## 1. Introduction

At present, the proportion of the elderly population in China is increasing, and the incidence of senile diseases is also increasing [1]. Osteoarthritis is a common chronic disease in the elderly. The clinical and pathological manifestations include hyperosteogeny and cartilage degeneration. The older the patient is, the higher the incidence is [2]. Total knee arthroplasty (TKA) can effectively improve the quality of life of patients on the basis of improving their physiological function and relieving pain, but there are many postoperative complications, including deep vein thrombosis (DVT) of the lower limbs, postoperative cognitive dysfunction, prosthesis loosening, and patellar arthritis [3]. The postoperative cognitive dysfunction can cause cognitive and social dysfunction or personality-acquired defects in patients, which are mainly manifested in the decline of attention, thinking ability and memory, as well as the decline of clinical social and activity ability, which have a great impact on the later life of the elderly [4]. The pathogenesis of postoperative cognitive dysfunction is complex, and some studies have shown that it may be related to the postoperative inflammatory response of the body. Surgical trauma can cause stress reaction in patients, release a large number of proinflammatory factors, and lead to and promote the occurrence and development of inflammatory reaction, involving the central nervous system of elderly patients, further affecting their cognitive function [5]. The formation of DVT refers to abnormal coagulation of deep vein blood and obstruction of lumen, which leads to venous reflux disorder. The clinical manifestations are pain, swelling of lower limbs, superficial varicose veins, and some systemic reactions such as increased body temperature [6]. Most of the thrombosis occurs in the braking state. For the elderly patients, the blood flow is slow, and they also need to be fixed or limited in local or whole body after the operation, which makes them more prone to thrombosis. If not handled properly, emboli can easily fall off, causing pulmonary embolism, which is life-threatening [7]. There are many reasons for deep vein thrombosis after TKA operation, among which age, obesity, bone cement use, and osteoarthritis are the most common ones. It has been reported in literature that anesthesia is also one of the factors that cannot be ignored [8]. Different anesthesia methods will have different effects on the coagulation function of patients. Therefore, we need to actively select the appropriate anesthesia methods in clinical to maintain a stable perioperative coagulation function. In this study, TKA patients were compared with general anesthesia and epidural anesthesia, and the influence of different anesthesia methods on perioperative cognitive function and deep vein thrombosis was discussed.

The article "Comparison of the Effects of Epidural Anesthesia and General Anesthesia on Perioperative Cognitive Function and Deep Vein Thrombosis in Patients Undergoing Total Knee Arthroplasty" was retracted in 2023. Reasons: unreliable results or conclusions; concerns about the data; concerns about the peer review; concerns about the citations.

## 2. Data and Methods

### 2.1. General Information

Total of 68 patients undergoing TKA in our hospital from September 2019 to March 2021 were selected, including 32 patients of unilateral knee replacement and 36 patients of bilateral knee replacement. Among them, there were 52 patients of primary disease, 9 patients of rheumatoid arthritis, and 7 patients of other diseases. According to different anesthesia methods, the patients were divided into the control group under general anesthesia and the observation group under epidural anesthesia, with 34 patients in each group. This study was approved by the hospital ethics committee, and informed consent was obtained from patients and their families.

### 2.2. Inclusion Criteria

(1) Presurgery color Doppler ultrasound or other examinations show no DVT formation in both lower limbs; (2) no severe heart, liver, kidney, and other organ diseases are combined; (3) ECG is normal; (4) normal coagulation function and platelets; and (5) no varicose veins in the lower limbs.

### 2.3. Exclusion Criteria

(1) Coagulation disorders, venous thrombosis, and a history of vascular surgery; (2) patients with severe dysfunction of the liver, heart, and kidney; and (3) patients with malignant tumor.

### 2.4. Anesthesia Method

TKA was selected into two groups, and the doctors, anesthesiologists, and nurses in the same group performed the operation. After entering the operating room, the vein was opened, and dynamic ECG, central venous pressure monitoring, and pulse oximetry monitoring were performed. At the same time, measure the bispectrum values. For the control group, general anesthesia was performed with rapid intravenous induction using midazolam 0.05 mg/kg, propofol 1.5 mg/kg, fentanyl 3 *μ*g/kg, and atracurium cissulfonate 0.2 mg/kg, as induction drugs, and tracheal intubation was conducted after the completion of anesthesia induction. Sevoflurane, atracurium cis-besylate, remifentanil, and propofol were selected for anesthesia maintenance during the operation, and the drug dose was adjusted according to the specific situation of patients.

The article "Comparison of the Effects of Epidural Anesthesia and General Anesthesia on Perioperative Cognitive Function and Deep Vein Thrombosis in Patients Undergoing Total Knee Arthroplasty" was retracted in 2023. Reasons: unreliable results or conclusions; concerns about the data; concerns about the peer review; concerns about the citations.

In the observation group, epidural anesthesia was adopted. A parallel tube was inserted through the space between the L2-3 and 3 lumbar spines. After successfully inserting the catheter, place the catheter about 3 cm toward the side of the head. Then, 8–20 mL of 2% lidocaine was infused through the catheter. According to the specific requirements of the patient's anesthesia plane, it was determined whether additional anesthetics were needed during the operation.

After successful anesthesia, the knee joint of the patient was slightly flexed, and the incision was made from the front of the patella to the medial side of the tibial tubercle. The operation was performed through the medial side of patella. The artificial knee joint was fixed with bone cement, and antibiotics were used prophylactically during the perioperative period. Anticoagulant drugs were given conventionally, and elastic bandages were used for 48–72 h.

### 2.5. Observation Indicators

The mean arterial pressure (MAP), heart rate (HR), and blood oxygen saturation (SpO_2_) were observed immediately before anesthesia (T1), 30 min after anesthesia (T2), after surgery (T3), and 1 d after surgery (T4). At T1 and T4, 2 mL fasting venous blood was drawn, and 0.13 moI/L sodium citrate was used for 9 : 1 anticoagulation. Then, the samples were centrifuged at 3000 r/min for 10 min to obtain the plasma to be tested. The coagulation functions of all patients at different time points were detected by the blood coagulation analyzer, including the changes of coagulation indexes such as platelets (PLC), fibrinogen (Fbg), prothrombin time (PT), and activated partial thrombin time (APTT).

The Montreal Cognitive Assessment Scale (MoCA) was used to assess the cognitive function of patients in two groups before surgery, 1 d and 3 d after surgery. The MoCA scale included 8 items in total, including visual space and executive function, naming, memory, attention, language, abstraction, delayed memory, and orientation. The total score was 30 points, and the educational year was ≤12 years plus 1 point. Patients with the total score less than 26 points were considered to have cognitive function impairment.

The article "Comparison of the Effects of Epidural Anesthesia and General Anesthesia on Perioperative Cognitive Function and Deep Vein Thrombosis in Patients Undergoing Total Knee Arthroplasty" was retracted in 2023. Reasons: unreliable results or conclusions; concerns about the data; concerns about the peer review; concerns about the citations.

The blood samples of the two groups were collected preoperatively, 1 d and 3 d after surgery, and the levels of brain-derived neurotrophic factor (BDNF) and nerve growth factor (NGF) in the peripheral blood of the two groups were measured by ELISA.

The number of postoperative mental disorders and DVT in the two groups was calculated. Psychiatric disorders criteria: (1) cognitive turbidity with time, place, and orientation disorders, inability to effectively concentrate attention, and confusion frequently occurring in daily events and activities; (2) susceptible to stimulation, improper behavior, cowardice, and overexcitation. Insanity or obvious signs of psychosis such as hallucinations, paranoia, and susceptibility; (3) physical disturbance is usually manifested as frequent walking back and forth. In a short period of time, there are contradictions, unable to correctly organize their own thinking, speech chaos, often with obvious language ambiguity, speed too fast, the creation of new words, aphasia errors, or language pattern disorder. One or more of the above symptoms can determine the existence of mental disorders.

### 2.6. Statistical Method

All data were analyzed by SPSS 19.0 statistical software, and measurement data were expressed as mean standard deviation. One-way analysis of variance was used for comparison between groups, and repeated measures analysis of variance was used for comparison at different time points. The count data were expressed as the rate (%) using the *χ*^2^ test. *P* < 0.05 indicated that the difference was statistically significant.

## 3. Result

### 3.1. Comparison of Clinical Data between the Two Groups

There was no significant difference in gender, age, bodyweight, education year, surgery time, and anesthesia time between the two groups (*P* > 0.05), as given in Table 1.

### 3.2. Changes of Hemodynamic Indexes in Two Groups

The MAP and HR of T4 in both groups were lower than those at T1, T2, and T3. The MAP of T2, T3, and T4 in the observation group was lower than that of the control group (*P* < 0.05), and there was no significant difference in HR between the two groups (*P* > 0.05). There was no significant change in SpO_2_ of T1–T4 in either group, and there was no significant difference between the two groups (*P* > 0.05), as shown in Figure 1.

### 3.3. Changes of Coagulation Indexes in Two Groups

There was no significant difference in PLC, Fbg, PT, and APTT of T1 between the two groups (*P* > 0.05). The PLC, Fbg, and PT of T4 in the observation group were not significantly different from those of T1 (*P* > 0.05), and APTT was lower than that of T1 (*P* < 0.05). The PLC, PT, and APTT of T4 in the control group were lower than those of T1 (*P* < 0.05), and there was no significant difference between Fbg of T1 (*P* > 0.05). The PLC, Fbg, and PT of T4 in the observation group were higher than those of the control group, and APTT was lower than that of the control group, and the differences were statistically significant (*P* < 0.05), as shown in Figure 2.

The article "Comparison of the Effects of Epidural Anesthesia and General Anesthesia on Perioperative Cognitive Function and Deep Vein Thrombosis in Patients Undergoing Total Knee Arthroplasty" was retracted in 2023. Reasons: unreliable results or conclusions; concerns about the data; concerns about the peer review; concerns about the citations.

### 3.4. Changes of MoCA Scores in Two Groups

There was no significant difference in MoCA scores before surgery between the two groups (*P* > 0.05). The MoCA scores of the two groups were lower than those of before surgery and 1 d and 3 d after surgery (*P* < 0.05). The scores of MoCA of the observation group were higher than those of the control group 1 d and 3 d after surgery, and the differences were statistically significant (*P* < 0.05), as shown in Figure 3.

### 3.5. Changes of BDNF and NGF Levels in Two Groups

There was no significant difference in BDNF and NGF before surgery between the two groups (*P* > 0.05). The BDNF and NGF of the two groups were lower than those before surgery and 1 d after surgery (*P* < 0.05). The BDNF and NGF levels in the observation group on 1 d and 3 d after surgery were higher than those in the control group, and the differences were statistically significant (*P* < 0.05), as shown in Figure 4.

### 3.6. Comparison of Postoperative Mental Disorders and DVT Incidence between the Two Groups

The incidence of postoperative mental disorders (2.94%) and DVT (2.94%) in the observation group was lower than those in the control group (29.41% and 26.47%), and the differences were statistically significant (*P* < 0.05), as shown in Figure 5.

## 4. Discussion

With the improvement of people's living standard and the advancement of joint surgery technology, the new materials and processes of artificial joints are continuously improved, and the use of artificial joints is becoming more and more common [9]. At present, TKA has been widely used in the clinical treatment of knee osteoarthritis. Knee replacement and active functional exercise after surgery can help patients to reduce joint pain, improve joint function, and correct joint deformities, thereby improving the quality of life [10, 11]. However, TKA is a highly difficult orthopedic operation, which has extremely high requirements for the surgeon, the operating room environment, surgical team, and sterility level, and it is easy to cause various complications [12]. A variety of trauma, pain, and surgical procedures can cause stress response of the body and change the endocrine function of the body, so that patients secrete a large amount of adrenal hormone. As an inducer of platelet aggregation, adrenal hormone can spontaneously activate platelets and increase the sensitivity and aggregation function of platelets. Especially in elderly patients undergoing joint replacement, under the influence of age, all functions will be degraded and the coagulation function will be decreased. In addition, surgical trauma will have a great impact on the body, easily leading to changes in patients' perioperative coagulation function [13–15]. The change of coagulation function is one of the pathological bases of DVT.

The article "Comparison of the Effects of Epidural Anesthesia and General Anesthesia on Perioperative Cognitive Function and Deep Vein Thrombosis in Patients Undergoing Total Knee Arthroplasty" was retracted in 2023. Reasons: unreliable results or conclusions; concerns about the data; concerns about the peer review; concerns about the citations.

TKA patients are mostly the elderly, and the anesthesia methods used are general anesthesia and epidural anesthesia. The drugs used in general anesthesia have a certain influence on coagulation function, and epidural anesthesia also has a certain influence on coagulation. Different anesthetic methods have different effects on coagulation function [16]. In order to maintain a good coagulation function in patients, we need to do a lot of work. Among them, different anesthesia methods will have different effects on the coagulation function of patients. Therefore, we need to actively select the appropriate anesthesia methods in clinical to maintain a stable perioperative coagulation function. The results of this study showed that, with the prolongation of anesthesia time, the hemodynamic MAP and HR of the two groups showed a downward trend. However, the improvement of blood flow in the observation group was better. At the same time, the coagulation indexes such as PLC, Fbg, PT, and APTT after operation made the patients in the observation group recover faster. It indicated that epidural anesthesia had less influence on hemodynamics and coagulation function of patients, thus reducing the incidence of DVT [17].

Epidural anesthesia makes anesthetics enter the patient's circulatory system through the epidural space, which reduces platelet activity, thus reducing the activation of blood coagulation. At the same time, it can also improve the deformation ability of red blood cells to a certain extent, effectively reducing the blood viscosity and avoiding the formation of venous thrombosis. However, general anesthesia played a certain role in activating platelet membrane glycoprotein, which might induce platelet activation. In addition, general anesthesia also has some influence on the endocrine system of patients undergoing surgery. At the same time, due to the decrease of the cardiovascular system function of elderly patients, they are sensitive to drugs and have a strong stress reaction, which may trigger platelet hyperfunction, resulting in hypercoagulable state of blood in patients during the perioperative period, leading to adverse reactions such as DVT [18].

The article "Comparison of the Effects of Epidural Anesthesia and General Anesthesia on Perioperative Cognitive Function and Deep Vein Thrombosis in Patients Undergoing Total Knee Arthroplasty" was retracted in 2023. Reasons: unreliable results or conclusions; concerns about the data; concerns about the peer review; concerns about the citations.

Studies have shown that elderly patients with TKA have a high probability of cognitive dysfunction during the perioperative period (3.5%–6.0%), which is mainly due to the poor physical condition and fragile physiological function of the nervous system in the elderly. Therefore, under the stimulation of anesthesia, it is easy to cause damage to the nervous system, which leads to cognitive dysfunction [19]. Patients with mild cognitive dysfunction can self-heal in a short time, but still can have different degrees of impact on life and work. Severe cognitive dysfunction will permanently lose social interaction and the ability to live independently. It has been reported in the literature that cognitive dysfunction during the perioperative period of TKA can indirectly induce senile dementia and improve the mortality after surgery [20]. Therefore, the selection of reasonable anesthesia has become an important part in improving the prognosis of patients with TKA. The results of this study showed that the MoCA scores of the observation group were higher than those of the control group 1 d and 3 d after operation, and the BDNF and NGF were higher than those of the control group. The levels of BDNF, NGF, and other neurotrophic factors can effectively promote the growth, proliferation, and differentiation of nerve cells in patients and can quickly repair the damaged nerve cells caused by surgical stimulation and other stimulations. It could be seen that epidural anesthesia had less effect on the postoperative mental state and neurotrophic factors, which was beneficial to the recovery of the patient [21, 22].

The results of this study also showed that the incidence of postoperative mental disorders and DVT in the observation group were lower than those in the control group. These results indicated that epidural anesthesia could effectively inhibit central sensitization and reduce the damage of intraoperative stress response to cognitive function. At the same time, it can reduce the hypercoagulable state of patients' blood and the probability of adverse reactions such as DVT.

In summary, epidural anesthesia for patients with TKA achieves better clinical effects, maintains stable hemodynamic and coagulation states, reduces stress response of patients, and reduces perioperative cognitive dysfunction and the incidence of DVT.

## Figures and Tables

**Figure 1:** Changes of hemodynamic indexes in two groups. *Note*. Compared with T4, ^*∗*^*P* < 0.05; compared with the control group, ^#^*P* < 0.05.

**Figure 2:** Changes of coagulation indexes in two groups. *Note*. Compared with T1, ^*∗*^*P* < 0.05; compared with the control group, ^#^*P* < 0.05.

The article "Comparison of the Effects of Epidural Anesthesia and General Anesthesia on Perioperative Cognitive Function and Deep Vein Thrombosis in Patients Undergoing Total Knee Arthroplasty" was retracted in 2023. Reasons: unreliable results or conclusions; concerns about the data; concerns about the peer review; concerns about the citations.

**Figure 3:** Changes of MoCA scores in two groups. *Note*. Compared with before surgery, ^*∗*^*P* < 0.05; compared with the control group, ^#^*P* < 0.05.

**Figure 4:** Changes of BDNF and NGF levels in two groups. *Note*. Compared with before surgery, ^*∗*^*P* < 0.05; compared with the control group, ^#^*P* < 0.05.

**Figure 5:** Comparison of postoperative mental disorders and DVT incidence between the two groups. *Note*. Compared with the control group, ^*∗*^*P* < 0.05.

**Table 1:** Comparison of clinical data between the two groups.

Group	Male/female	Age (years)	Body mass (kg/m^2^)	Education year (years)	Surgery time (min)	Anesthesia time (min)
Control group (*n* = 34)	19/15	58.92 ± 5.59	32.16 ± 6.16	10.28 ± 3.95	94.32 ± 21.52	116.59 ± 29.86
Observation group (*n* = 34)	21/13	59.05 ± 6.02	31.85 ± 7.03	11.13 ± 3.81	97.59 ± 22.07	118.19 ± 30.91
*t/χ* ^2^ value	0.243	0.125	0.193	0.903	0.619	0.217
*P* value	0.622	0.901	0.847	0.370	0.538	0.829

## Data Availability

The data used and/or analyzed during the current study are available from the corresponding author.
